# Effects of Afatinib on Development of Non-Small-Cell Lung Cancer by Regulating Activity of Wnt/*β*-Catenin Signaling Pathway

**DOI:** 10.1155/2022/5213016

**Published:** 2022-06-28

**Authors:** Yue Wu, Jiajing Zhang, Changping Yun, Chenchen Dong, Ye Tian

**Affiliations:** Second Department of Respiratory Medicine, The Second Affiliated Hospital of Qiqihar Medical College, Qiqihar, 161001 Heilongjiang, China

## Abstract

Lung cancer has been one of the deadliest cancers in the world. Afatinib is an ErbB family irreversible blocker that was authorized by the FDA and EMA in 2013 for the treatment of advanced EGFR mutation-positive NSCLC. Therefore, we aim to discover the impact of Afatinib on the development of non-small-cell lung cancer (NSCLC) via modulating the Wnt/*β*-catenin signaling pathway. The objective remission rate (ORR), disease control rate (DCR), progression-free survival (PFS), and overall survival (OS) in 22 patients with clinical NSCLC were analyzed as follow-up targets after Afatinib therapy. The differences between the effects of Afatinib treatment and DDP+PEM treatment for conventional chemotherapy were used to measure NSCLC cell proliferation by CCK-8 assay; then those on NSCLC apoptosis were measured by flow cytometry. Patients who received Afatinib had better ORR, DCR, PFS, and OS than those in the conventional chemotherapy group. Meanwhile, CCK-8 assay shows that the number of colony formation of NSCLC cells after Afatinib treatment was less than that in the DDP+PEM group. And NSCLC apoptosis was higher than that in the DDP+PEM group. Phenomenologically, experimental results show that Afatinib can affect the behaviors of NSCLC cells. After treating NSCLC cells with Afatinib, the protein expressions of three serum tumor markers (CEA, CA125, and CY-FRA21-1) were detected by Western blotting, with the findings indicating that the protein expressions in NSCLC cells treated with Afatinib were lower than those of the DDP+PEM group, which indicates that Afatinib treatment can reduce the expressions of tumor markers, and inhibit the development of tumors. Afatinib can affect the progression of NSCLC by modulating the Wnt/*β*-catenin signaling pathway's activity as a new potential therapeutic drug for NSCLC.

## 1. Introduction

Nowadays, lung cancer has been the deadliest cancer [1]. In the United States, lung cancer is the first cause of cancer death, with a 5-year survival rate of barely 15% [2]. Non-small-cell lung cancer (NSCLC) is a specific pathological form of lung cancer, accounting for 85% of all cases. NSCLC includes multiple types of cancers, such as lung adenocarcinoma (LUAD), lung squamous carcinoma (LUSC), and large cell lung cancer [3]. Over the past few years, the treatment of NSCLC has been developed into targeted therapy and immunotherapy [4]. Although the emergence of immunotherapy has played an essential role in the treatment of patients with NSCLC, identifying driver mutations and treating them individually can often produce long-lasting effects while sustaining a high standard of living [5].

The development of drug therapy for NSCLC is relatively rapid, which has been reported that the treatment of Anamorelin can improve the weight and symptom burden in patients with NSCLC and anorexia [6]. SNH, the active component of Houttuynia cordata, can inhibit the transfer of NSCLC cells [7]. The five types of TCM, namely, terpenoids, flavonoids, polysaccharides, natural polyphenols, and alkaloid monomers, can have significant inhibitory effects on NSCLC [8]. Cell lines that express high EGFR undergo receptor-mediated apoptosis [9]. And other reports have shown that Afatinib inhibited the survival of NSCLC cell lines, H23 and H292 [10], and Afatinib's inhibitory effects on the development of NSCLC have been confirmed.

ErbB receptor family, also known as the EGF receptor family or I-receptor family, includes epidermal growth factor receptor (EGFR) or ErbB1/Her1, ErbB2/Her2, ErbB3/Her3, and ErbB4/Her4 [11], overexpresses, or mutates in many malignancies particularly in breast cancer, ovarian, and NSCLC. Excessive expression and activation are linked to a poor prognosis, cancer metastasis, and a shorter life expectancy [12]. EGFR is a glycoprotein with a transmembrane domain, one of the four members of tyrosine kinase receptor ErbB family. Its signal cascade reactions include proliferation, differentiation, and division of cells, as well as a key regulator in survival and cancer development [13], with activation associated with multiple human cancers. Furthermore, there is a lot of research that confirmed that a combination of EGFR tyrosine kinase inhibitor (TKI) and ethanedioic acid (EA) can induce necrosis and cell cycle stasis of breast cancer cells and inhibit Wnt/*β*-catenin signal transduction [14]. Therefore, for cancer chemotherapy, inhibition of EGFR is one of the most important targets [15]. Inhibitors acting on EGFR tyrosine kinase are the gold standard of therapy for EGFRM+NSCLC patients [16]. It has been reported that Afatinib has clinical activity against NSCLC with rare and complex EGFR mutations [17]; it improves progress free survival (PFS), time to failure (TTF), and objective response rate (ORR) [18]. Compared with a similar drug, Gefitinib, Afatinib has better effects on untreated patients who have EGFR mutations in NSCLC [19].

Afatinib (BIBW 2992, USA: Gilotrif™, other countries: Giotrif©) is an ErbB family irreversible blocker that was authorized by the FDA and EMA in 2013 for the treatment of advanced EGFR mutation-positive NSCLC [20]. Besides, it has been reported that Afatinib can significantly improve progression-free life expectancy in patients who have head and neck squamous cell carcinoma (HNSCC) [21]. Moreover, the combination of Afatinib and Temozolomide can significantly inhibit the carcinogenicity of glioblastoma and delay the tumor development and progression in vivo [22]. The pathogenesis of NSCLC is related to Wnt/*β*-catenin. At the same time, the therapeutic effect of Afatinib on NSCLC has been confirmed. However, there are few reports on the specific treatment methods of Afatinib on NSCLC.

Therefore, this study combined current information and resources to deeply explore the relationship between Afatinib and Wnt/*β*-catenin. We discussed the treatment effects of Afatinib as a targeted drug for EGFR mutations in NSCLC. And we used Afatinib as a targeted drug for the treatment of NSCLC and thoroughly investigated the regulatory effect of Afatinib on the development of NSCLC. In addition, we analyzed the objective remission rate (ORR), disease control rate (DCR), progression-free survival (PFS), and overall survival (OS) in 22 patients with clinical NSCLC.

## 2. Experimental Methods

### 2.1. Clinical Research Subjects

All patients have signed informed consent before receiving medication, with administration and follow-up approved by the Ethics Committee of the Second Affiliated Hospital of Qiqihar Medical College. The primary goal of this research is to investigate the statistical influence of Afatinib on ORR, DCR, PFS, and OS in patients' prognoses.

The study comprised 50 patients with early nonsmoking lung cancer. The 50 patients underwent radical surgical treatment from the Second Affiliated Hospital of Qiqihar Medical College. The 50 patients were all EGFR mutation-positive and were clinically diagnosed as NSCLC. The inclusion criteria include early nonsmoking lung adenocarcinoma, aged over 18 years, and lung cancer stages IIIB/IV that had not yet been pathologically confirmed. Among the subjects, 22 patients were treated with Afatinib after operation, and another 28 patients were treated with chemotherapeutic drugs DDP+PEM. All 50 patients were free from other drugs' influence, with the median 41.6-month follow-up period for at least 80 times.

### 2.2. Cell Culture

H460 cells in NSCLC cell line were cultivated in Dulbecco's modified Eagle medium (DMEM) which contained 10% fetal bovine serum with 100 *μ*IU/mL penicillin and 100 *μ*IU/mL streptomycin and then transferred into the sterile incubator containing 5% CO_2_ at 37°C for further culture. The cells were used in the following drug induction experiments. The density reached 70%~80% at the moment.

### 2.3. Drug Treatment

All the 50 subjects treated with drugs were given the same adjuvant therapy of radiotherapy and chemotherapy. Among them, 22 patients were administrated with 40 mg/day of Afatinib and 28 patients were treated with DDP+PEM, to reflect the drug effects by measuring the size and diameter of tumors with imaging according to Version 1.1 of Response Evaluation Criteria for Solid Tumors (RECIST v1.1).

#### 2.3.1. H460 Administration

Afatinib was dissolved in DMSO. Lung cancer cells in logarithmic phase were seeded into a six-hole plate and pretreated with 8 *μ*M Afatinib or DMSO as control.

### 2.4. CCK-8 Assay

NSCLC cells were cultivated into the culture plate with 96 holes, which was divided into three groups, including the Afatinib group, the control group: DDP+PEM, and the normal saline group. After administration correspondingly, 10 *μ*L CCK-8 (Beyotime Institute of Biotechnology, Beijing, China) was put in each hole and cultivated at 37°C for 2 hours. The absorbance values were measured at 450 nm with Tecan Infinite M200 Micro Plate Reader (LabX, Switzerland), expressing the corresponding optical density ratio as cell viability.

### 2.5. Flow Cytometry

About 2 × 10^5^ NSCLC cells were digested with trypsin in each group and collected in a 1.5 mL EP tube and, then to remove trypsin, centrifuged at 2000 g/min for 5 minutes. After the supernatant has been removed, to keep the cells suspended, 500 *μ*L binding buffer was added, and 5 *μ*L Annexin V-FITC was added to incubate in the dark for 30 minutes. Then, 5 *μ*L propidium iodide (PI) was lightly commixed then cultured 5 minutes at room temperature. The total number of cells in Q2 and Q3 quadrants was tested with Annexin-V-FITC detection kit (K201-100, BioVision, USA) and flow cytometry (version 10.0, FlowJo, FACS Calibur™, BD, USA).

### 2.6. Western Blotting

We used 1% Triton lysis buffer to dissolve the cells. Finally, the samples were separated by preprepared SDS-PAGE electrophoresis after adding protein loading buffer, and then, the gel was transferred to PVDF membrane for Western blotting analysis. PGSK3*β* (sc-81495) was purchased from Santa Cruz Biotechnology, USA. *β*-Catenin (bs: 1165R), Cyclin D1 (bs: 20596R), and Goat Anti-rabbit IgG (bs: 0295G) were purchased from Bioss (China, Beijing). MiniChemi™ 500 small chemiluminescence imaging and analysis device were used to process Western blotting images. (Sage Creation Science, Beijing, China).

### 2.7. ELISA

Patients' fasting blood samples were taken before receiving any cancer treatment, which were centrifuged at 3000 rpm for 10 minutes to obtain serum. CEA, CYFRA21-1, and CA125 were detected by ELISA with TECAN and kit (IDL Biltech, Sweden).

### 2.8. Statistical Analysis

The protein gray scale of Western blotting was scanned by ImageJ (1.4.3.67 Broken symmetry software), and the Kaplan-Meier method was used to control the survival curve. All the data were analyzed by GraphPad Prism 7.0 Software (GraphPad Software, La Jolla, CA, USA). The mean and standard deviation (SD) were used to express all of the variables, and multiple groups were compared through ANOVA. *P* < 0.05 was thought to be significant statistically.

## 3. Results

### 3.1. Afatinib Can Improve the Poor Prognosis of Patients with NSCLC

To compare the effects of Afatinib treatment on the prognosis of NSCLC patients, 22 patients who received Afatinib were followed up randomly, and their ORR, DCR, PFS, and OS were analyzed statistically. The results showed that ORR, DCR, PFS, and OS in the Afatinib group were much greater compared with the DDP+PEM group, indicating that Afatinib can be considerably enhanced the prognosis of NSCLC patients and their health status. As a result, Afatinib has a good therapeutic effect on NSCLC, which needs further development and demonstration. See Table 1 and Figure 1. Through a randomized follow-up of 50 patients with NSCLC treated with Afatinib and conventional DDP+PEM, Afatinib can improve the prognosis of patients with NSCLC, and ORR, DCR, PFS, and OS can also be improved (Figure 1), without unexpected adverse events during administration.

### 3.2. Afatinib Is Closely Related to the Proliferation of NSCLC Cells

To further verify the therapeutic impact of Afatinib on patients with NSCLC, NSCLC cells were cultured and divided into three groups: the Afatinib group, the control group, and DDP+PEM, and the saline group. CCK-8 assay was used to test the impact on Afatinib medication on NSCLC cell growth. As shown in Figure 2, the results showed that after Afatinib treatment, the colony formed by cell proliferation was far less than that in the DDP+PEM group and saline group, indicating that Afatinib can stop NSCLC cells from proliferating. Figure 2 shows that Afatinib showed significant antiproliferative activity against NSCLC.

### 3.3. Effects of Afatinib on Apoptosis of NSCLC Cells

Since the treatment of Afatinib can stop NSCLC cells from proliferating, the effects of Afatinib on NSCLC apoptosis were discovered using Annexin-V-FITC/PI staining. When the apoptosis rates in Q2 and Q3 quadrants were counted, it was found that the apoptosis in Q2 and Q3 quadrants of NSCLC cells treated with Afatinib was far higher than those in DDP+PEM group and saline group, indicating that Afatinib can increase NSCLC apoptosis, promote the apoptosis, and inhibit the proliferation of NSCLC cells.  Figure 3 shows that Afatinib promoted NSCLC apoptosis suggesting that the treatment of NSCLC by Afatinib may have blocked the progression of NSCLC cell cycle by binding Afatinib to EGFR mutant receptors.

### 3.4. Effects of Afatinib on Protein Expression of Three Serum Tumor Markers

The above results showed that Afatinib can stop NSCLC cells from proliferating and accelerate NSCLC apoptosis. And then how the molecular effects affect the development of NSCLC was verified by the following experiments. The expressions of CEA, CYFRA21-1, and CA125 in serum of patients in the Afatinib and DDP+PEM groups were detected by ELISA. The findings revealed that the positive rate of CEA, CYFRA21-1, and CA125 in control group (*P* < 0.05) was much higher compared with the group in the serum of Afatinib (Table 2). The changes in the protein expressions of three serum tumor markers (CEA, CA125, and CY-FRA21-1) were detected by Western blotting. As shown in Figure 4, after treatment with Afatinib, the protein expressions of CEA, CA125, and CY-FRA21-1 in NSCLC cells were lower than that in DDP+PEM and saline groups, indicating that Afatinib can reduce the expressions of tumor markers, inhibit the growth of tumors, and improve the health status of patients with NSCLC.

### 3.5. Effects of Afatinib on Proliferation of NSCLC Cells by Regulating Wnt/*β*-Catenin Signaling Pathway

The above shows Afatinib can stop NSCLC cells from proliferating and accelerate their apoptosis, which can also interfere with the expressions of tumor markers, so it can be concluded that Afatinib can treat NSCLC and alleviate the poor prognosis of patients with NSCLC. To further verify the effects of Afatinib, the effects of different drug treatments on the activity of Wnt/*β*-catenin signaling pathway and the protein expression of Cyclin D1 were discovered by Western blotting. As shown in Figure 5, the protein expressions of *β*-catenin and P-GSK3*β* in NSCLC cells treated with Afatinib were lower than those in the DDP+PEM group or saline group, and the protein expression of Cyclin D1 decreased. Therefore, the inhibitory effects of Afatinib on the proliferation of NSCLC cells are reached by regulating the activity of Wnt/*β*-catenin signaling pathway.

## 4. Discussion

Afatinib, a tyrosine kinase inhibitor, is a widely used drug for NSCLC [23]. The current inhibitor of EGFR mutations in NSCLC has emerged as one of the most common treatments for advanced or metastatic NSCLC [24]. Moreover, Afatinib-treated patients have been shown to have a prolonged PFS [25], which was consistent with our conclusion. After NSCLC cells were treated with three different drugs (Afatinib, DDP+PEM, and saline), the sensitivity of NSCLC to the three drugs was detected. And this effect on proliferation was associated with apoptosis. However, how Afatinib mediates apoptosis by regulating EGFR still needs further exploration. Carcinoembryonic antigen (CEA) is an effective biomarker for the diagnosis of primary hepatic carcinoma (PHC) and metastatic hepatic carcinoma (MHC) [26], which was expressed as the occurrence of cancers. In the typing of ovarian cancer, the expression of CA125 in II-type ovarian cancer (advanced stage) was significantly higher than that in I-type. Tumor biomarker CA125 can be used as a major marker for ovarian cancer [27], and serum tumor markers, carcinoembryonic antigen (CEA), cancer antigen 125 (CA125), and cytokeratin 19 segments (CYFRA21-1) can all be used to monitor the response of patients with NSCLC to chemotherapy or targeted therapy [28]. Afatinib also inhibited protein expressions of three serum tumor markers more strongly than that in DDP+PEM and saline groups (Figure 4), indicating that the expressions of tumor markers in NSCLC cells treated with Afatinib decreased, inhibiting the recurrence and occurrence of tumors. We speculated that the regulatory effects of Afatinib on the expressions of tumor markers are also associated with EGFR mutations in NSCLC. Serum tumor indicators have been linked to EGFR mutations, combined with other clinical factors, enhancing the ability to distinguish EGFR mutations in patients [29].

The Wnt/*β*-catenin signaling pathway has anything to do with the occurrence and development of cancer. It is also involved in the development of NSCLC. According to previous research, through the Wnt/-catenin signaling pathway, PMMB-317 stopped A549 cells from migrating with dose-dependence, blocked G2/M cell cycle, induced apoptosis, and inhibit the activity of EGFR [30], which were consistent with our speculation that the effects of Afatinib on NSCLC cells can be mediated by inhibition of EGFR receptor activity. However, whether Afatinib can act on the development process of NCSLC through the Wnt/*β*-catenin signaling pathway has not been mentioned. On this basis, we further explored its mechanism. We detected the activity changes of Wnt/*β*-catenin pathway in NSCLC cells treated with Afatinib with Western blotting. It turned out that the activity of pathway proteins, *β*-catenin and p-GSK3*β*, was inhibited after treatment with Afatinib, as well as Cyclin D1 expression, which means that Afatinib can affect the proliferation of NSCLC cells through Wnt/*β*-catenin pathway. A specific mechanism could be explained by the fact that Afatinib inhibits EGFR receptor activity, and EGFR inactivation inhibits the activity of Wnt/*β*-catenin signaling pathway.

## 5. Conclusions

This study verified the regulatory relationship between Afatinib and the Wnt/*β*-catenin signaling pathway and explained Afatinib can affect the process of NSCLC through the Wnt/*β*-catenin signaling pathway. It offers experimental proof and basis for further research on non-small-cell lung cancer and the treatment mechanism of Afatinib. Above these results, it is concluded that Afatinib can inhibit the activity of EGFR receptors. The activity of WNT/*β*-catenin signaling pathway would also be inhibited after the inhibition of EGFR, which ultimately affects the proliferation and apoptosis of NSCLC cells. This study adds to the body of evidence supporting Afatinib's use in the treatment of NSCLC. However, there are still some limitations in our study. Our study used 50 patients as the dataset and studied a few variables. Thus, we need to explore more data.

## Figures and Tables

**Figure 1:** Effects of Afatinib and routine treatment on PFS and OS in patients with NSCLC.

**Figure 2:** Effects of Afatinib on proliferation of NSCLC cells detected by CCK-8. Effects of different drug treatment groups on the proliferation of NSCLC cells detected by CCK-8 assay. Experimental group: Afatinib group; control groups: DDP+PEM and saline group; *n* = 5; ^∗^*P* < 0.05.

**Figure 3:** Effects of Afatinib on NSCLC apoptosis detected by flow cytometry. This figure counts the number of cells in Q2 and Q3 quadrants to reflect the apoptosis. Experimental group: Afatinib group; control groups: DDP+PEM group and saline group; *n* = 5; ^∗^*P* < 0.05.

**Figure 4:** Effects of Afatinib on protein expressions of tumor markers. Effects of Afatinib on the occurrence of tumors detected by Western blotting. After treating NSCLC cells with three drugs, the difference between protein expressions of three tumor markers was compared. Experimental group: Afatinib group; control groups: DDP+PEM group and saline group; *n* = 5; ^∗^*P* < 0.05.

**Figure 5:** Effects of Afatinib on the activity of Wnt/*β*-catenin signaling pathway. Effects of different drugs on proteins related to the Wnt/*β*-catenin signaling pathway detected by Western blotting. Experimental group: Afatinib group; control groups: DDP+PEM group and saline group; *n* = 5; ^∗^*P* < 0.05.

**Table 1:** Effects of Afatinib on ORR and DCR in 22 patients.

Systemic tumor response to treatment (*n* = 22)	
ORR, % (95% CI)	38.4 (15.2, 59.3)
DCR, % (95% CI)	78.5 (60.8, 97.8)
Complete response, *n* (%)	0 (0.0)
Partial response, *n* (%)	8 (35.7)
Stable disease, *n* (%)	12 (57.4)
Progressive disease, *n* (%)	5 (15.9)

Kaplan-Meier analysis on 22 patients treated with Afatinib and conventional DDP+PEM for the relationship between Afatinib and prognosis, ORR, and DCR in patients with NSCLC.

**Table 2:** Expression of tumor markers in serum.

Indicators	Afatinib	DDP+PEM	*P*
LDH (U/L)	136.00 (34.00)	181.00 (57.00)	<0.001
CEA (*μ*g/L)	2.40 (5.42)	5.60 (28.65)	<0.001
CYFRA21-1 (ng/mL)	1.14 (1.23)	2.78 (3.67)	<0.001
CA125 (U/mL)	4.98 (12.21)	31.24 (78.56)	<0.001

## Data Availability

The datasets used and/or analyzed during the present study are available from the corresponding author on reasonable request.
